# Puerarin Attenuates LPS-Induced Inflammatory Responses and Oxidative Stress Injury in Human Umbilical Vein Endothelial Cells through Mitochondrial Quality Control

**DOI:** 10.1155/2021/6659240

**Published:** 2021-02-27

**Authors:** Xing Chang, Tian Zhang, Dong Liu, Qingyan Meng, Peizheng Yan, Duosheng Luo, Xue Wang, XiuTeng Zhou

**Affiliations:** ^1^State Key Laboratory of Dao-di Herbs, National Resource Center for Chinese Materia Medica, China Academy of Chinese Medical Sciences, Beijing, China; ^2^Guang'anmen Hospital, Chinese Academy of Traditional Chinese Medicine, Beijing, China; ^3^Shandong University of Traditional Chinese Medicine, Jinan, Shandong, China; ^4^Institute of the History of Chinese Medicine and Medical Literature, China Academy of Chinese Medical Sciences, Beijing, China; ^5^Institute of Chinese Medicine, Guangdong Pharmaceutical University, Guangzhou, China; ^6^School of Business Macau University of Science and Technology, Taipa, Macau, China

## Abstract

Atherosclerosis is closely associated with the inflammatory reaction of vascular endothelial cells. Puerarin (Pue), the main active component isolated from the rhizome of *Pueraria lobata*, is an isoflavone compound with potent antioxidant properties. Although Pue exhibits promising antiatherosclerotic pharmacological effects, only a few studies have reported its protective effect on endothelial cells. This study found that Pue could partly regulate mitochondrial function in human umbilical vein endothelial cells (HUVECs) and reduce or inhibit lipopolysaccharide-induced inflammatory reactions and oxidative stress injury in HUVECs, likely via mitochondrial quality control. Furthermore, the protective effect of Pue on HUVECs was closely related to the SIRT-1 signaling pathway. Pue increased autophagy and mitochondrial antioxidant potential via increased SIRT-1 expression, reducing excessive production of ROS and inhibiting the expression of inflammatory factors and oxidative stress injury. Therefore, Pue may improve mitochondrial respiratory function and energy metabolism, increasing the vulnerability of HUVECs to an inflammatory state.

## 1. Introduction

Atherosclerosis (AS) is a protective response to arterial wall endothelium and smooth muscle injury, including the formation of lipid streaks and fiber injury, and is always accompanied by an inflammatory reaction [1, 2]. When the inflammatory response is excessive, it may trigger vascular endothelial cell damage and plaque formation [3, 4]. Endothelial cell structure and function play important roles in maintaining a balance of microcirculation and smooth blood flow, especially in AS development [5, 6]. Endothelial cells are the main cells constituting the intima of the artery wall and are the barrier between blood and external tissues. They function to regulate blood flow, vascular tension, antithrombotic and procoagulant activities, and lipoprotein metabolism [7]. Endothelial cells also produce cytokines and can regulate immune responses through their barrier and secretion functions [8]. Furthermore, endothelial cells can secrete bioactive substances, such as nitric oxide (NO) and endothelin, and affect the function of smooth muscle cells, platelets, and white blood cells [9].

Endothelial cell injury and dysfunction are involved in the early initiation of AS [10]. For instance, during the early stage of AS, endothelial cells can produce a series of inflammatory factors that may further aggravate endothelial cell dysfunction, participate in thrombosis, and promote the occurrence and development of AS [11]. During the state of inflammatory stress, endothelial cell function and gene expression switch from a resting to an activated state, contributing to various inflammatory reactions [12]. Endothelial cells may be affected by inflammatory factors produced by other cells and can also affect the proliferation and contraction of smooth muscle cells through paracrine signaling [13]. The proliferation of smooth muscle cells is an important feature of late AS development [14].

Most studies to date have focused on the role of endothelial dysfunction in vasculitis and microcirculation diseases. With respect to these types of diseases, endothelial dysfunction caused by inflammation is more likely to lead to AS [15, 16]. During the development of AS, inflammatory reactions are often related to reactive oxygen species- (ROS-) mediated oxidative stress [17]. With the occurrence and development of inflammation, increased activated infiltrating immune cells, and inflammatory resident cells, the demand for mitochondrial energy gradually increases, leading to hypoxia and mitochondrial quality control (MQC) disorder. Furthermore, ROS are overproduced, and endothelial cells exhibit more severe oxidative damage [18, 19].

Mitochondria are the powerhouse of oxidative phosphorylation in eukaryotes [20], wherein carbohydrates, fats, and proteins are oxidized and catabolized to produce energy [21, 22]. Pyruvate is hydrolyzed to form triacyl acid and pyruvic acid in the mitochondria. Ultimately, H_2_O and CO_2_ are generated, and adenosine triphosphate (ATP) is released to sustain physiological cell functions [23]. Studies have shown that mitochondrial involvement is an important link in AS progression [24]. Mitochondrial energy metabolism disorder is one of the early indications of vascular endothelial cell dysfunction [25]. During AS progression, mitochondrial energy metabolism disorder mainly manifests as respiratory dysfunction and decreased expression of energy metabolism-related genes and proteins [26]. Mitochondria are important mediators in cells, and mitochondrial dysfunction can indirectly activate a variety of inflammatory signal transduction pathways, leading to tissue and cell damage. ROS-mediated oxidative stress may result in MQC disorder through direct cytotoxicity and can promote the occurrence and development of local inflammatory responses [27].

Oxidative stress and inflammation are interdependent, especially in mitochondria. Excessive ROS production at inflammatory sites can lead to oxidative stress-induced damage to mitochondria. Mitochondrial ROS and the accompanying products of oxidative stress can synergistically enhance the response of inflammatory factors. Mitochondria may be the “Trojan horse” of inflammation while maintaining basic cell function [28]. In addition, a study by Chen revealed that damaged mitochondria activate inflammatory bodies of NLR family pyrin domain containing 3 (NLRP3) [29]. Furthermore, activation of NLRP3 is inhibited when mitochondrial autophagy clears abnormal mitochondria and damaged proteins [30]. The oxidative effect of mitochondrial ROS on mitochondrial DNA during activation of NLRP3 leads to a partial inflammatory potential of free circulating mitochondrial DNA. This shows that oxidative stress and the mitochondrial pathway can affect MQC and endothelial cell inflammatory responses in an interdependent manner.

Puerarin (Pue) is the main active component of *Pueraria lobata*, which is used in traditional Chinese medicine. Pue is a flavonoid glycoside extracted from the dried roots of *P*. *lobata* [31, 32]. Because of its noticeable estrogen-like effects, Pue helps treat atherosclerotic diseases and protect endothelial cell function [33]. Pue also significantly reduces lipopolysaccharide- (LPS-) induced p-NF-kappa B-p65 and Bax expression and increases the expression levels of Bcl-2. Furthermore, Pue can inhibit the release of inflammatory cytokines and protect umbilical vein endothelial cells [34]. Other studies have shown that Pue can reduce vascular endothelium injury and the expression of IL-1*β*, IL-8, ICAM-1, and PAI-1 in the supernatant of human umbilical vein endothelial cells (HUVECs) stimulated with LPS. It can also reduce LPS-induced neutrophil adhesion to HUVECs, inhibiting LPS-induced endothelial injury [35].

Although experimental studies have confirmed that Pue has a significant protective effect on endothelial cells, the specific mechanism remains unclear. In the current study, we investigated whether the inhibitory effect of Pue on LPS-induced endothelial cell inflammation and oxidative stress injury was mediated by mitochondria.

## 2. Results

### 2.1. Pue Improved HUVEC Activity in LPS-Induced Inflammation

A HUVEC inflammatory model was established by stimulating HUVECs with LPS to preliminarily confirm the effect of Pue on the function of HUVECs in an LPS-mediated inflammatory state. Different concentrations of Pue (10 mg/L, 20 mg/L, 50 mg/L, 100 mg/L, and 150 mg/L) were then used as intervention treatments. HUVEC activity was determined using CCK-8 assays. CCK-8 analysis showed that LPS decreased the activity of HUVECs compared with that in the control group, as shown in Figure 1(a). Pretreatment with different Pue concentrations improved HUVEC vitality after LPS treatment, with the cell activity being most significant after pretreatment with 100 mg/L Pue (Figure 1(b)). Accordingly, 100 mg/L Pue was chosen as the optimal drug concentration to treat HUVECs in subsequent experiments. The analysis also showed that LPS increased apoptosis levels of HUVECs, but 100 mg/L Pue inhibited the apoptosis (Figures 1(c) and 1(d)). These results indicated that Pue maintained the activity of HUVECs and inhibited cell apoptosis under an LPS-induced inflammatory state.

### 2.2. Pue Inhibited LPS-Induced Inflammatory Responses and Oxidative Stress Damage in HUVECs

We found that Pue could also reduce LPS-induced inflammatory injury. Compared with that in the control group, the LPS-induced expression of inflammatory factors, TNF-*α*, and IL-18 was significantly increased in HUVECs treated with LPS (Figures 2(b) and 2(c)). Furthermore, the expression level of the anti-inflammatory factor IL-10 was significantly reduced (Figure 2(a)). Pretreatment of HUVECs with Pue reversed the LPS-induced increase in TNF-*α*/IL-18 levels and downregulation of the IL-10 expression (Figure 2(a)–2(c)). The results confirmed that Pue intervention could improve the HUVEC inflammatory response induced by LPS.

We further investigated the protective mechanism of Pue in improving the vitality and reducing the vulnerability of HUVECs under LPS-induced inflammation. To explore the protective effect of Pue on the redox state of endothelial cells and mitochondrial oxidative stress damage, enzyme-linked immunosorbent assays (ELISAs) were used to evaluate the activity of antioxidant enzymes, such as glutathione (GSH), superoxide dismutase (SOD), and glutathione peroxidase (GPx). We found that the inflammatory state induced by LPS exhibited reduced GSH, SOD, and GPx activity in HUVECs (Figures 3(d)–3(f)). Pretreatment of the cells with Pue resulted in increased GSH, SOD, and GPx activity (Figures 3(d)–3(f)). These results suggested that LPS-induced inflammation could induce oxidative stress damage by inhibiting the activity of antioxidant enzymes, including GSH, SOD, and GPx. However, Pue was able to reverse this phenomenon, which further confirmed the pharmacological activity of Pue against oxidative stress.

### 2.3. Pue Regulated HUVEC MQC under LPS-Induced Inflammation

Mitochondria are the main sites of ATP production that are required for cellular energy metabolism. Studies have demonstrated that LPS-induced inflammatory responses can cause severe damage to the structure and function of mitochondria [36, 37]. In the current study, we evaluated HUVECs for mitochondrial ROS generation levels and mitochondrial membrane potential (MMP). Compared with those in the control group, the level of mitochondrial ROS generation was increased (Figures 4(a) and 4(f)), and the MMP levels were significantly reduced (Figures 4(d) and 4(e)). Pue treatment of HUVECs resulted in significantly increased MMP levels (Figures 4(d) and 4(e)), while the mitochondrial ROS generation levels were significantly reduced (Figures 4(a) and 4(f)).

Mitochondria are the main sites of oxygen consumption in cells and the main ROS source as well as the main target of ROS attack. Excessive production of mitochondrial ROS results in the release of proinflammatory factors IL-18 and TNF-*α* and directly affects mitochondrial structure and function [38–40]. LPS-induced HUVEC inflammatory responses and oxidative stress damage changed the structure and function of mitochondria compared with those in the control and destroyed the MMP. However, Pue intervention significantly increased the activity and number of mitochondria, restored the MMP, and inhibited mitochondrial ROS generation. We also evaluated mitochondrial respiratory complexes I and III activity by ELISA (Figures 4(b) and 4(c)). Mitochondrial respiratory complexes I and III showed reduced expression under LPS-induced inflammatory injury, but their activities were restored with Pue intervention.

### 2.4. Pue Promoted HUVEC Mitochondrial Energy Metabolism under LPS-Induced Inflammation

Abnormal mitochondrial energy metabolism and respiratory function are closely related to mitochondrial dysfunction [41–43]. In the current study, we investigated whether Pue under inflammatory conditions could improve mitochondrial energy metabolism levels and respiratory function in HUVECs using a mitochondrial energy metabolism test. Compared with those from the control group, HUVECs treated with LPS exhibited significant reduction in mitochondrial respiration levels (Figure 4(a)), maximum respiration capacities (Figure 4(b)), spare respiratory capacities (Figure 4(c)), and ATP production capacities (Figure 4(d)); nonmitochondrial oxygen respiration level (Figure 4(e)) and proton leakage (Figure 4(f)) increased significantly. However, Pue pretreatment reversed all these reductions, resulting in significant increases in the level of mitochondrial energy metabolism and respiratory function (Figures 4(a)–4(d)), the level of nonmitochondrial oxygen respiration (Figure 4(e)), and proton leakage values (Figure 4(f)) was inhibited.

To investigate how Pue improved the mitochondrial respiratory function of HUVECs in an inflammatory state, EX-527 was used, which is an effective and specific inhibitor of sirtuin-1 (SIRT-1). The results showed that mitochondrial respiratory function of HUVECs was significantly inhibited in the EX-527 + LPS + Pue group compared to that in the LPS + Pue group (Figures 4(a)–4(f)). This demonstrated that the effect of Pue on improving mitochondrial respiratory function was eliminated by the SIRT-1 inhibitor EX-527. Pue was able to improve mitochondrial respiratory function of LPS-treated HUVECs and protect the mitochondria and HUVECs. According to the results, the protective mechanism of Pue may have been mediated through SIRT-1.

### 2.5. Pue Regulated HUVEC Autophagy in an Inflammatory State through Sirt-1

The protective mechanism of Pue against oxidative stress injury and mitochondrial function damage in HUVECs was further explored. Expression levels of select mRNAs were detected by real-time quantitative polymerase chain reaction (qPCR). The qPCR analysis showed that the mRNA levels of atg3, atg7, sirt-1, and PINK1/parkin were significantly lower in the LPS group compared to those in the control group, but they were significantly higher in Pue + LPS-treated HUVECs (Figures 5(a)–5(e)). The mRNA levels of atg5, atg7, sirt-1, and PINK1/parkin in HUVECs treated with EX-527 + Pue + LPS were also significantly reduced. However, the mRNA levels of atg5, atg7, sirt-1, and parkin were significantly increased in HUVECs treated with the SIRT-1 activator SRT1720 (SRT1720 + Pue + LPS). Transmission electron microscopy showed that LPS treatment significantly inhibited mitochondrial autophagy, and Pue increased the level of mitochondrial autophagy (Figure 5(f)). As shown in Figures 5(g) and 5(h), the protein expression of Sirt-1, LC3-I\II, Beclin-1, and Bcl-2 decreased significantly in the LPS group but increased significantly in the LPS + Pue group. However, when ex527 was used, the effect of Pue on autophagy was eliminated. However, srt1720 could restore and improve the autophagy regulation ability of Pue. These results suggested that Pue regulated autophagy through the SIRT-1 signaling pathway.

### 2.6. Inhibition of the SIRT-1 Signaling Pathway Abolished Pue-Mediated Protection

To further determine whether Pue could induce mitochondrial and HUVEC protection through the SIRT-1 signaling pathway, we used EX-527 and SRT1720 to intervene in Pue + LPS-treated HUVECs. The specific regulatory mechanism of Pue was verified through evaluation of cell viability, apoptosis levels, antioxidant enzyme activity, anti-inflammatory ability, and mitochondrial function in the various HUVEC groups. As shown in Figure 6(a), CCK-8 revealed that EX-527 treatment significantly reduced the activity of HUVECs treated with Pue + LPS. Besides, EX-527 treatment eliminated the protective effect of Pue on the mitochondria of HUVECs treated with LPS as well as the inhibitory effect of Pue on the inflammatory response and oxidative stress injury (Figures 6(b)–6(j)). Meanwhile, SRT1720 eliminated the ability of Pue to regulate the inflammatory reaction and oxidative stress injury of HUVECs (Figures 6(b)–6(j)). Laser scanning confocal images of myosin-VI also showed that the expression of myosin-VI was rapidly decreased and increased by LPS and Pue, respectively; EX-527 can eliminate the regulatory effect of Pue, and SRT1720 can further restore the regulatory effect of Pue (Figure 6(k)). These results confirmed that Pue improved the mitochondrial activity of HUVECs and inhibited LPS-induced inflammatory responses and oxidative stress injury through SIRT-1.

## 3. Discussion

Inflammation and oxidative stress are the main risk factors of cardiovascular damage in patients with AS. Pue, a natural antioxidant, can play a key role in regulating inflammatory responses and oxidative stress injury. However, few studies are aimed at revealing the underlying mechanism by which Pue reduces endothelial cell vulnerability to inflammatory conditions. In the current study, we found that an LPS-induced inflammatory response in HUVECs led to increase ROS production in mitochondria and greater MQC disorder and aggravated the damage caused by oxidative stress. Pue regulates MQC, enhances mitochondrial autophagy, and inhibits LPS-induced inflammation and oxidative stress injury in HUVECs. Pue also increased the MMP and energy metabolism of the HUVECs, increased the activity of SOD and other antioxidant kinases, inhibited the excessive ROS production and inflammation-induced oxidative stress damage, weakened the LPS-induced inflammatory response, and reduced HUVEC vulnerability to the inflammatory state.

Furthermore, it was found that intervention with EX-527, a selective SIRT-1 inhibitor, counteracted Pue regulation of MQC and the protective effect of Pue on HUVECs. However, intervention with the SIRT-1 activator SRT1720 restored the protective effect of Pue to normal or even higher than normal levels. Accordingly, we conclude that Pue protected HUVECs from inflammation through SIRT-1. These results indicate that Pue, as a natural antioxidant, regulated MQC through the SIRT-1 signaling pathway and reduced the vulnerability of HUVECs to the inflammatory state.

Damage to endothelial cells due to changes in membrane structure leads to the production of antiarterial antibodies and the activation of the complement system, which aggravates vascular endothelial damage and promotes AS development [44]. Cytokinins, inflammatory factors, and mitochondrial dysfunction in the environment can all regulate the activity and function of endothelial cells by changing the extracellular concentration of oxidative stress products [45, 46]. A large number of aging vascular endothelial cells are present in advanced arterial plaques. In cell aging, mitochondria dysfunction intensifies, and the level of intracellular ROS significantly increases. The abnormally elevated ROS in the cell further induces vascular damage during cell aging and aggravates lesions [47].

In the current study, we found that markers related to oxidative stress were significantly upregulated in HUVECs treated with LPS, while the expression of mitophagy-related genes and antioxidant stress kinases was significantly downregulated. This indicated that inflammation could increase oxidative stress injury and inhibit mitophagy. Under oxidative stress injury, mitochondrial folding of proteins and useless organelles could not be cleared in a timely manner because mitophagy was inhibited, and the normal level of energy metabolism and respiratory chain function of the mitochondria may have been disrupted, resulting in a rapid decrease of mitochondrial activity and MQC disorder. MQC is an important mechanism for eukaryotes to maintain a relatively stable number and function of mitochondria [48]. MQC ensures the normal operation of the mitochondrial network, further regulates the timely updating of mitochondria, and maintains the relative stability of the quantity and quality of mitochondria in endothelial cells, or it may participate in the occurrence and development of AS [49, 50].

The distribution of mitochondria in endothelial cells can also affect cell signal transduction. Under physiological conditions, endothelial cell mitochondrial dynamics are in a state of stable dynamic equilibrium [51, 52]. Inflammation-induced perinuclear aggregation of mitochondria can lead to mitochondrial ROS accumulation and affect the transcription level of the vascular endothelial growth factor gene [49]. Main functions of mitochondria in endothelial cells are transmitting cell response to environmental signals and participating in the protective mechanism of endothelial cells under oxidative stress and inflammation [53–55].

Many natural products of plants can protect endothelial cells by regulating mitochondrial function and reducing endothelial cell vulnerability under stress [56, 57]. Our study directly confirmed the protective mechanism of natural antioxidants on endothelial cells through MQC. We also found that Pue could regulate the mitophagy of endothelial cells and maintain normal cell activity. Autophagy/mitophagy not only controls the homeostasis of blood vessels but also functions in mitochondria energy metabolism and the mitochondrial antioxidant system to maintain the basic physiological functions of mitochondria [56, 57]. Further research is needed to determine the mechanistic interaction between autophagy/mitophagy and oxidative stress in the inflammatory state. Furthermore, the mechanism by which Pue affects mitochondrial quality by regulating autophagy levels remains unclear.

SIRT-1 is a highly conserved NAD^+^-dependent histone deacetylase. In recent years, SIRT-1 has been shown to play important roles in many biological processes, including cell differentiation, aging, apoptosis, physiological rhythm, metabolic regulation, transcription regulation, signal transduction, and oxidative stress [58, 59]. SIRT-1 exists in the nucleus and is highly expressed in vascular endothelial cells. Moreover, the serum SIRT-1 level in patients with cardiovascular disease is significantly higher than that in healthy individuals [60, 61]. EX-527 is an effective selective inhibitor of SIRT-1 and is often used to block the regulation of SIRT-1. We found in the current study that EX-527 could counteract the protective effect of Pue in HUVECs. However, on intervention with SRT1720, the protective effect of Pue on HUVECs was restored, as along with its regulatory effect on MQC. These results indirectly confirmed that Pue regulated autophagy in HUVECs through SIRT-1 and may further protect HUVECs from inflammatory responses and oxidative stress injury. However, animal studies will be needed to confirm whether Pue directly affects blood flow and AS by regulating MQC and endothelial cells through SIRT-1.

In conclusion, we found that cell viability and MQC of HUVECs were regulated through the SIRT-1 signaling pathway. LPS treatment reduced SIRT-1 signaling and induced oxidative stress injury and apoptosis. Pue was able to regulate MQC by upregulating SIRT-1 signaling, improving the level of autophagy in HUVECs, and further reducing the vulnerability and oxidative stress injury of HUVECs under inflammatory conditions. It should be noted that this study examined only whether Pue improves oxidative stress injury of HUVECs by regulating MQC in an inflammatory state. The results do not imply Pue can also exert the same protective effect on HUVECs under other stress conditions (such as high glucose and hypoxia).

Notwithstanding this limitation, hypoxia and high glucose stress are related to oxidative stress and MQC disorder. This study characterized Pue as a natural antioxidant; further clinical and basic studies will confirm the regulatory mechanism of Pue on MQC and oxidative stress. In the future, Pue may be developed as a candidate drug for the clinical treatment of AS. We expect Pue to become a treatment strategy potentially widely used to treat a variety of cardiovascular diseases.

## 4. Materials and Methods

### 4.1. Cell Culture and Treatment

HUVECs were purchased from the Institute of Basic Medicine, Chinese Academy of Medical Sciences (Beijing, China). LPS was acquired from Sigma-Aldrich (St. Louis, MO, USA). SRT1720 and EX-527 were purchased from MedChemExpress (Princeton, NJ, USA). Pue (purity ≥ 98%) was purchased from the Chinese Medicine Resource Center, Chinese Academy of Traditional Chinese Medicine (Beijing, China).

The cells were cultured in Dulbecco's modified Eagle's medium (DMEM, Gibco, Carlsbad, USA) containing 10% fetal bovine serum (Gibco) and 100 *μ*g/mL penicillin-streptomycin (Gibco). Cells were passaged using trypsin-EDTA (Gibco). The cells were incubated at 37°C, 95% humidity, and 5% CO_2_. The medium was renewed every 2 days. HUVECs were used up to passage five [62]. The HUVECs were activated with 10 *μ*g/mL LPS for 24 h [63] and pretreated with 10, 20, 50, 100, or 150 mg/L Pue for 24 h before LPS induction. As indicated, HUVECs were incubated with EX-527 (MedChemExpress) for 6 h to inhibit SIRT-1 activity or with SRT1720 (MedChemExpress) for 6 h to activate SIRT-1.

### 4.2. CCK-8 Assays

HUVECs were determined to be in good condition, with a total cell coverage rate of more than 90%. The cells were washed with phosphate-buffered saline (PBS, Gibco) and then digested with trypsin. The digestion was terminated by adding fresh complete DMEM, and the cells were then counted. The cells were seeded into 12-well plates (50,000 cells/well) and incubated for 12 h. The medium was discarded, the cells were rinsed twice with PBS, and the adherent cells were then observed under an inverted microscope (Olympus, Tokyo, Japan). Cellular metabolic activity as an indicator of cell viability was measured by the CCK-8 essay.

### 4.3. Mitochondrial Membrane Potential (MMP)

MMP of the HUVECs was measured using JC-1 Dye (MedChemExpress). HUVECs were washed three times with PBS and then stained with JC-1 Dye for 30 min in a dark room. The HUVECs were then washed three times with PBS, and the mitochondrial membrane potential images were captured using a Nikon A1 laser confocal microscope (Nikon, Chiyoda, Japan).

### 4.4. Laser Confocal Microscopy

HUVECs were fixed with 4% paraformaldehyde for 10 min, washed with PBS three times, and blocked on ice with PBS for 30 min. The HUVECs were then incubated with primary antibody (myosin-VI, Abcam, Cambridge, UK) against Tom20 at 4°C overnight. After washing with PBS three times, the cells were stained with Alexa fluor-594-conjugated goat anti-mouse secondary antibody in 1% BSA/PBS at 4°C for 1 h. Nuclei were stained with 4′,6-diamidino-2-phenylindole (DAPI), and images were captured using a Nikon A1 confocal microscope.

### 4.5. ELISA Quantitative Analysis

The cells were digested with 0.25% trypsin in PBS according to the manufacturer's instructions. The SOD, GSH, GPx, IL-10, IL-18, and TNF-*α* contents were detected using a total assay kit.

### 4.6. Quantitative Real-Time PCR

Total RNA was isolated from HUVECs using a Quick-RNA Microprep Kit (Zymo Research, Irvine, CA, USA). An iScript cDNA Synthesis Kit (Bio-Rad, Hercules, CA, USA) was used to reverse transcribe 150–250 ng total RNA into complementary DNA (cDNA). The cDNA samples were diluted 10-fold with ddH_2_O, and real-time quantitative PCR (qPCR) was performed on a LightCycler 480 Instrument using 2 *μ*L cDNA. Relative gene expression was calculated using the 2^−*ΔΔ*Ct^ method [64].

### 4.7. Cellular Respiration Assays

An XFp Extracellular Flux Analyzer (Seahorse Biosciences, North Billerica, MA, USA) was used according to the manufacturer's instructions to analyze the oxygen consumption rate (OCR) of intact cells in real time. Briefly, HUVECs were inoculated at 5 × 10^5^ cells/well. The results were normalized to the actual cell count determined immediately after obtaining the OCR recording.

### 4.8. Statistical Analysis

All statistical analyses were performed using the Statistical Product and Service Solutions (SPSS) 22.0 software package (IBM Corp., Armonk, NY, USA) and GraphPad Prism version 7.0 (GraphPad Software, San Diego, CA, USA). All data are expressed as mean ± SEM and were evaluated by analysis of variance; *p* < 0.05 was considered statistically significant. The normal distribution of the data was confirmed by Shapiro–Wilk test.

## Figures and Tables

**Figure 1:** Pue improves the activity of human umbilical vein endothelial cells (HUVECs) under LPS-induced inflammation. (a) Cell viability in an LPS-induced inflammatory state was determined using the CCK-8 method. After LPS stimulation, HUVEC viability was severely reduced. (b) HUVEC treatment with Pue at different concentrations (10, 20, 50, 100, and 150 mg/L). HUVEC viability under different drug concentrations was determined using the CCK-8 method. (c, d) HUVEC apoptosis level was analyzed before and after Pue administration. ^∗^*p* < 0.05.

**Figure 2:** Pue inhibits LPS-induced inflammatory responses and oxidative stress damage in human umbilical vein endothelial cells (HUVECs). (a–f) Proinflammatory and anti-inflammatory factors and antioxidant enzymes were evaluated using ELISA. ^∗^*p* < 0.05.

**Figure 3:** Pue improves mitochondrial activity under LPS-induced inflammation and oxidative stress damage. (a, f) HUVEC mitochondrial ROS expression. (d, e) Detection of mitochondrial membrane potential. (b, c) ELISA detection of mitochondrial respiratory complex I and III activity. ^∗^*p* < 0.05.

**Figure 4:** Pue promotes mitochondrial energy metabolism in human umbilical vein endothelial cells (HUVECs) induced with LPS: (a) basic mitochondrial respiratory level; (b) maximum respiratory capacity; (c) spare respiratory capacity; (d) ATP production capacity; (e) nonmitochondrial oxygen respiration; (f) proton leakage level. ^∗^*p* < 0.05.

**Figure 5:** Mechanism of Pue in regulating mitochondrial autophagy through SIRT-1. (a–e) Changes in transcription of atg3, atg7, sirt-1, and PINK1/parkin were determined by qPCR. ^∗^*p* < 0.05. (f) Mitochondrial autophagy was observed with transmission electron microscopy. (g, h) Protein expression of Sirt-1, LC3-I\II, Beclin-1, and Bcl-2 was measured using western blotting. ^∗^*p* < 0.05.

**Figure 6:** Inhibition of the SIRT-1 signaling pathway abolishes Pue-mediated protection. (a) CCK-8 analysis in different groups of human umbilical vein endothelial cells (HUVECs). (b–j) Enzyme-linked immunosorbent assays (ELISAs) showed antioxidant enzyme activities and anti-inflammatory factors in the different groups. (k) Laser confocal scanning was used to observe the alterations of myosin-VI in endothelial cells under Pue treatment. ^∗^*p* < 0.05.

## Data Availability

The data used to support the findings of this study are available from the corresponding author upon request.
